# Accuracy combining different brands of implants and abutments

**DOI:** 10.4317/medoral.18137

**Published:** 2012-12-10

**Authors:** María F. Solá-Ruíz, Eduardo Selva-Otaolaurruchi, Gisela Senent-Vicente, Inés González-de-Cossio, Vicente Amigó-Borrás

**Affiliations:** 1 Adjunt Professor. Department of Buccofacial Prosthetics, Faculty of Medicine and Dentistry, Universitat de València, Spain; 2 Titular Professor. Department of Buccofacial Prosthetics, Faculty of Medicine and Dentistry. Universitat de València, Spain; 3 Associate Professor. Department of Buccofacial Prosthetics, Faculty of Medicine and Dentistry. Universitat de València, Spain; 4 Chairman of Materials. Department of Mechanical and Material Engineering. Polytechnic University of Valencia, Spain

## Abstract

Objective: To evaluate the vertical misfit between different brands of dental implants and prosthetic abutments, with or without mechanical torque, and to study their possible combination. Study design: Five different brands of implant were used in the study: Biofit (Castemaggiore, Italy), Bioner S.A. (Barcelona, Spain), 3i Biomet (Palm Beach, U.S.A.), BTI (Alava, Spain) and Nobel Biocare (Göteborg, Sweden), with standard 4.1 mm heads and external hexagons, and their respective machined prosthetic abutments. The implant-to-abutment fit/misfit was evaluated at four points (vestibular, lingual/palatine, mesial and distal) between implants and abutments of the same brand and different brands, with or without mechanical torque, using SEM micrographs at 5000X. Image analysis was performed using NIS-Elements software (Nikon Instruments Europe B.V.). Results: Before applying torque, vertical misfit (microgaps) of the different combinations tested varied between 1.6 and 5.4 microns and after applying torque, between 0.9 and 5.9 microns, an overall average of 3.46±2.96 microns. For manual assembly without the use of mechanical torque, the best results were obtained with the combination of the 3i implant and the BTI abutment. The Nobel implant and Nobel abutment, 3i-3i and BTI-BTI and the combination of 3i implant with BTI or Nobel abutment provided the best vertical fit when mechanical torque was applied. Conclusions: The vertical fits obtained were within the limits considered clinically acceptable. The application of mechanical torque improved outcomes. There is compatibility between implants and abutments of different brand and so their combination is a clinical possibility.

** Key words:**Vertical fit, implant, prosthetic abutment, combination.

## Introduction

Restorative dentists tend to work with the products of one particular brand of implant system or another. However, there is an increasing demand for prosthodontic treatment from patients who already have unloaded maxillary implants. In such cases the dentist will have to choose between using the prosthetic components of the same brand as the patient’s implant(s) or using the brand that he/she is familiar with. If the first option is chosen, then the dentist will have to purchase the components and learn how to handle them, which will increase economic cost and treatment time. The second option is only possible if there is compatibility between implant and abutment.

There is a great deal of information on the clinical consequences of a bad fit between implant and prosthetic abutment (1-4). Discrepancies greater than 10 microns can have biological effects (bacterial microfiltration) (1,2) and produce inadequate mechanics (loosening and rotating screws) (3), which may lead to complete treatment failure. Values of 10 microns or less do not seem to have consequences for hard or soft tissues (4). The relationship between prosthetic abutments and the implants which support them has been studied for machined titanium and zirconia abutments, and for cast and premachined abutments (5). Nevertheless there is little published research on the combination of elements from different manufacturers (6).

The aim of this study was to analyze the vertical misfit (microgap) between implant external hexagons and prosthetic abutments of different brands, with and without the application of mechanical torque, and, if possible, their combination in clinical practice.

 The null hypothesis was that there is compatibility and the possibility of combining, without a loss of treatment quality, the five different brands of implants included in the present study (implants with standard 4.1 mm heads and external hexagons) and their respective machined prosthetic abutments.

## Study Design

Five titanium implants of five different brands were used in the study: Biofit (Castemaggiore, Italy), Bioner S.A. (Barcelona, Spain), 3i Biomet (Palm Beach, U.S.A.), BTI (Alava, Spain) and Nobel Biocare (Göteborg, Sweden), with external hexagons and 4.1 mm diameter platforms and their 25 corresponding machined titanium prosthetic abutments. Both implants and abutments were standard products freely available on the market and belonged to the same product batches.

Abutments were fitted onto implants of the same brand and onto implants from different manufacturers, examining microgaps or the degree of vertical misfit at the abutment-to-implant union. The systems were first assembled manually and evaluated, then evaluated a second time after applying a mechanical torque of 32Ncm.

Microgap measurements were performed using a scanning electron microscope (SEM), JEOL JSM 6300 (Tokyo, Japan).

For each implant/abutment assembly, four perimeter zones (mesial, lingual, distal and vestibular) were selected, taking micro-graphs of each at 5000X. In this way four images were obtained of each union. Three measurements of the microgap (microns) were made from each micrograph at the same points on each image, based on a line drawn arbitrarily on the first image which was then transferred onto the rest of the images (Fig. 1). Image analysis was performed using NIS-Elements software (Nikon Instruments Europe B.V.).

**Figure 1:** SEM image at 5000x showing the three lines, drawn arbitrarily, where measurements were taken.

Twenty five different implant/abutment combinations were tested, with and without mechanical torque, obtaining a total sample of 600 microgap measurements.

All values obtained underwent statistical analysis using the Mann-Whitney U test for two independent samples (combinations of similar quality) and box plots were produced to represent the distribution of continuous variables; the significance level was taken as 5% (p<0.05).

## Results

-Results without torque.

Implants and abutments were assembled manually without applying torque.

Figure 2 : The box graph represents the distribution of 300 microgap measurements made of the 25 possible implant/abutment combinations, 12 measurements per combination: Results covered a range of values that suggested that implant/abutment combinations could be classified as three types, which we will call excellent, good and acceptable. Excellent combinations are those whose interquartile range falls below the first quartile (1.6 microns); good combinations are those with an interquartile range between the first and third quartiles; acceptable are combinations that exceed the third quartile of 5.4 microns. These three groups of Implant/abutment combinations according to the quality of the fit were determined by applying descriptive concepts alone ( Table 1).

**Figure 2:** Combinations of all implants and all abutments without application of mechanical torque.

**Table 1:** Implant/abutment combinations without torque.

The BIOFIT implant in combination with any abutment and the BIOFIT abutment in combination with any implant produced the worst quality fit.

The Mann-Whitney non-parametric test was applied to each pairing of combinations, in which the variable measured is distributed so that it is statistically equivalent; this determined that the three best combinations were: 3iBiomet-BIONER, 3i-BTI and NOBEL-BTI. The remaining combinations, all good, were positioned on a second level.

-Results with torque.

In this second test, implants and abutments were assembled applying a mechanical torque of 32Ncm as recommended by the manufacturers.

Figure 3: The box graph represents the distribution of 300 microgap measurements made of the 25 possible implant/abutment combinations, 12 measurements per combination: combinations considered ‘excellent’ were those for which the interquartile range fell below the first quartile (0.9 microns); combinations considered ‘good’ were all those for which the interquartile range was between the first and third quartile; ‘acceptable’ combinations were those with an interquartile range exceeding 5.9 microns.

**Figure 3:** Combinations of all implants and all abutments with application of mechanical torque.

This data is shown in  Table 2. The BIONER-BIOFIT and BTI-3i combinations produced the lowest quality fit. When combinations of implants and abutments of the same brand were analyzed, the best results were achieved by Nobel B-Nobel B, with 100 % of measurements less than 2 microns; the worst combination was BIOFIT-BIOFIT that showed 50% of measurements higher than 6 microns.

**Table 2:** Implant/abutment combinations with torque.

 When the Mann-Whitney non-parametric test was applied to each combination pair with p-values greater than 0.05, in other words, those which follow similar distributions, it was found that BTI-BTI, 3i Biomet-3i Biomet and Noble B-Nobel B showed a statistically equivalent distribution.

## Discussion

Hypothesis was confirmed, as there is compatibility and possibility of combining the different brands of implants and their respective machined prosthetic abutments without a loss of treatment quality. There is a good deal of published research on fit and precision in implant and abutment manufacturing, whether machined or cast, but there is little to be found among the literature which examines the possibility and convenience of combining implants from one manufacturer with abutments from another.

There is clear agreement among authors that the exactitude of hexagon machining is crucial and significant differences have been detected between different manufacturers (7-9). The fabrication of implants and their related components should present a high degree of homogeneity. It has also been pointed out that many manufacturers fail to provide scientific information about products to their users (10).

Various authors have studied the fit of machined titanium abutments and others cast from different materials such as zirconia, concluding that machined titanium and zirconium oxide produce the best fit (11-13). For this reason, machined titanium components were chosen for this study.

Various techniques have been used to test fit/misfit, such as human observation of samples under magnification, measurement of cross-sections and impression techniques, among others (8,14). For this study, electron microscope measurement was chosen for its precision and simplicity, taking the precaution of maintaining the same positioning of samples and visual plane throughout the study (15).

The study evaluated vertical misfit, using the protocol followed by Holmes et al. (16) in his work, which, with torque, obtained values varying between 0 and 10 microns, an average of 3.17±2.73 microns. Kano et al. (17) report a vertical misfit of 5.6 ± 6.4 microns for machined abutments, these producing better results than cast or premachined elements. This author also found a considerable horizontal discrepancy, a problem that the present study has not evaluated. Tsuge et al. (18) measured vertical misfit, finding microgaps of between 2.3 and 5.6 microns, results that coincide with our own.

Measurements were performed in two stages; firstly evaluating implant/abutment combinations assembled using manual torque and secondly applying a torque of 32 Ncm as recommended by the manufacturers. It was shown that the use of mechanical torque produces a better fit in all cases (19,20).

In spite of the limitations of the present study it may be concluded that: The vertical fit observed in all cases fell within the limits of clinical acceptability.

The best results, in manual assembly without mechanical torque, were achieved by the combinations 3i Biomet and BTI abutment, 3iBiomet-BIONER and NOBEL-BTI; the worst combinations were with the Biofit implant and any abutment. When mechanical torque was applied the Nobel, 3i Biomet and BTI implants with their corresponding prosthetic abutments produced the best fit, together with the combinations of 3i Biomet implant with BTI or Nobel abutments.

The application of mechanical torque improved results.

There is compatibility between the implants and abutments of the different manufacturers tested and so their combination is a clinical possibility.
